This article has been retracted.

# Performance Evaluation of Knowledge Sharing in an Industry-University-Research Alliance Based on PSO-BPNN

**DOI:** 10.1155/2022/1283588

**Published:** 2022-05-10

**Authors:** Lin Wang

**Affiliations:** Graduate School, Jilin Jianzhu University, Changchun, China

## Abstract

Knowledge sharing performance is very important to evaluate the interests of industry university research alliance. Firstly, this paper puts forward the index system of knowledge sharing performance evaluation of industry university research alliance. A BP neural network (BPNN) and a PSO-improved BP neural network (PSO-BPNN) are used to establish the evaluation model, and the accuracy of the model is evaluated. The prediction accuracy is evaluated by comparing the predicted value with the target value. Through comparative analysis, it is found that the performance evaluation model based on PSO-BP neural network has high accuracy and applicability, and is an effective method of alliance knowledge sharing performance evaluation.

## 1. Introduction

An industry-university-research alliance (IURA) is a strategic alliance established among enterprises, universities, and research institutions as a systematic way to optimize resource allocation. In an era of accelerated scientific and technological progress and increasingly fierce market competition, IURAs represent a new form of strategic cooperation designed to enhance a country's independent innovation capacity. Through the strong combination and complementary resources of enterprises, universities, and research institutions, IURAs offer comprehensive advantages within the operation process, promote the upgrading of industrial structure, and strongly drive economic development. Knowledge sharing within an IURA is an effective way to promote cross-field cooperation, leverage the synergy and multiplier effects of knowledge dissemination and diffusion, and enhance the growth of organizational knowledge. As an important component of knowledge sharing, performance evaluations play a crucial role and should be highly valued. An evaluation of the knowledge sharing performance of an IURA can provide a theoretical basis for the alliance to improve its knowledge sharing methods.

The backpropagation (BP) neural network (BPNN) is an error BP training algorithm consisting of a set of artificial neural networks (NNs) referred to as the BP algorithm. The BPNN has a wide range of applications in research concerning performance evaluations. Cui proposed an NN-based knowledge transfer effectiveness evaluation method [1]. Wang and Guo used the BPNN method to construct a comprehensive evaluation model to assess the internal knowledge transfer performance of enterprises [2]. Zhuang and Guo establish the evaluation index system, and propose an improved algorithm model based on BP neural network [3]．

Li et al. proposed and applied an improved particle swarm optimization (PSO) algorithm-optimized FNN to corrosion detection in reinforced concrete with multisensor information fusion [4]. PSO-improved NNs have been widely used in the engineering field. Li et al. constructed a prediction model for electrical power substitution potential based on a gray relational analysis (GRA)-improved PSO-BP (GRA-IPSO-BP) [4]. Shang used the improved PSO model to optimize the BP neural network to identify psychological stress [5]．

In this paper, we propose that the knowledge sharing performance of an IURA can be evaluated using a BPNN improved with PSO. PSO-BPNN uses the characteristics of PSO algorithm to optimize the weight and threshold of BP neural network, which can get the weight and threshold closer to the global optimal solution, so as to overcome the disadvantage that BP neural network is easy to fall into the local optimal solution. An index system for evaluating the knowledge sharing performance of an IURA is first developed and then tested on enterprises to obtain performance evaluation data, which are used to train the PSO-BPNN. We use the PSO-BPNN to evaluate the knowledge sharing performance of an IURA. Compared with the evaluation value of the BPNN and the target value, the evaluation value of the PSO-BPNN features a relatively small error, which proves the accuracy of the method. The use of the PSO-BPNN to evaluate the knowledge sharing performance of an IURA can prevent the problems of slow error convergence and susceptibility to being trapped in local minima, thereby improving the accuracy of evaluations. Therefore, the optimization of the BPNN with the improved PSO algorithm reduces the prediction error of the BPNN and renders predicted values more practical, providing a reliable basis for IURAs to develop knowledge sharing policies.

## 2. Construction of the IURA Knowledge Sharing Performance Evaluation Index System

### 2.1. Selection of Evaluation Indices

#### 2.1.1. Indices of Knowledge Sharing Performance Evaluation

CNKI, Google Scholar, Emerald Insight, and ProQuest were searched with the keywords “knowledge sharing performance” and “knowledge management performance”; this search yielded 911 relevant articles. After screening, 27 articles closely related to knowledge sharing performance evaluating index systems were identified. The top 12 most frequently used knowledge sharing evaluation indices are shown in Table 1.

The existing findings on knowledge sharing performance indicate that researchers have analyzed the evaluation index systems of knowledge sharing performance according to the characteristics, objectives, and influencing factors of knowledge sharing. Their findings are reasonable, scientific, relevant, and offer important references for this study.

#### 2.1.2. Evaluation Index System for the Knowledge Sharing Performance of IURAs

In 1994, Teece proposed dynamic capability theory in Dynamic Capabilities of Firms: An Introduction and systematically elaborated this theory in Dynamic Capability and Strategy Management, which was published in 1997. Dynamic capability refers to the ability of a firm to integrate, construct, and reallocate its internal and external capabilities to respond to a dynamically changing competitive environment. The possession of resources and organizational capabilities alone is insufficient to maintain a competitive advantage in a dynamically changing competitive environment. Enterprises should continually develop and update their capabilities or acquire dynamic capabilities to exploit and update their resource and organizational capabilities [6]. An IURA is open to enterprises, universities, and institutes, and members can join or withdraw at any time. Such decisions are made according to the dynamic demands of participants and their performance after admission. As a result, the internal environment of an alliance changes dynamically. To exploit new knowledge and new resources, update their own capabilities and maintain a competitive advantage, alliance members must integrate internal resources and knowledge shared by other alliance members. The process by which alliance members absorb such knowledge and participate in joint development and innovation is called alliance collaboration. Dynamic capability theory fully explains the mechanism of IURAs, and the extent of members' dynamic capability determines the capacity for member collaboration. Since performance evaluation is associated with the expected targets and profits associated with participant cooperation, the performance evaluation indices of IURAs should motivate alliance members to participate in cooperation. The aims of enterprises and institutes participating in knowledge sharing within an IURA are to enhance their innovation ability and their ability to handle and adapt to changing external environments, to increase the added value of knowledge, and to maintain a competitive advantage. Therefore, IURA knowledge sharing performance evaluation indices should capture the capabilities of members and the value of their knowledge.

Performance evaluation is associated with the targets and profits the participants expect to realize through cooperation. Enterprises and institutes participating in IURA knowledge sharing aim to enhance their innovation ability and their ability to manage and adapt to changing external environments, to increase the added value of knowledge, and to maintain a competitive advantage. Therefore, IURA knowledge sharing performance evaluation indices should capture the capabilities of members and the value of their knowledge. Dynamic capability is also pivotal in maintaining the profitability of enterprises [7]. Thus, the concept of dynamic capability was introduced to evaluate the knowledge sharing performance of IURAs.

Teece defined dynamic capability along three dimensions: “perceiving and recognizing opportunities and threats,” “seizing opportunities,” and maintaining a competitive advantage by strengthening, combining, and protecting. Based on the findings of dynamic capability theory and given the existing research results on evaluation systems and the characteristics of IURAs, we built an IURA knowledge sharing performance evaluation system that incorporated the ability to identify opportunities, the ability to seize opportunities, the ability to revolutionize and integrate knowledge, and the added value of knowledge.

*(1) The ability to Identify Opportunities*. The internal environment of an IURA is dynamic and open, since new members can join the alliance at any time; thus, old and new members all face the same opportunities and challenges. Members who identify a development opportunity earlier are more likely to acquire knowledge and generate profits. Thus, the ability to identify new opportunities is the primary factor in knowledge sharing.

The knowledge leverage. The knowledge lever refers to the identification and sharing of knowledge resources in relatively competitive fields through as many methods and routes as possible [8].

The ability to perceive opportunities. An organization with the ability to perceive opportunities can identify and create opportunities through data collection and analysis. Since most new opportunities are undifferentiable, the ability to perceive opportunities is extremely critical for alliance members to maintain competitiveness and profits.

The ability to create opportunities. Alliance members should acquire enough detailed environmental information to take the initiative in creating opportunities for knowledge sharing. Such opportunities are created through investments in research activity, including investigations into the potential demands of customers, reassessments of technology, industry and market structure evolution, and examinations of competitor responses.

The ability to adapt. The ability to adapt refers to the capacity of alliance members to identify and use opportunities in emerging markets. Members with greater adaptability have more powerful dynamic capabilities [9].

*(2) The ability to Seize Opportunities*. The ability to seize opportunities refers to the capacity of alliance members to make decisions, facilitate mutual understandings among members, and formulate knowledge sharing schemes. Members should reach consensus, learn, acquire, share, absorb and interpret knowledge, and make efficient decisions to seize opportunities for development.

Reaching a consensus. A mutual understanding and consensus among alliance members is the key to evolutionary innovation and overcoming organizational inertia and a basis upon which members can collaborate and share knowledge.

Learning. Learning is the core element needed to create and update the dynamic capabilities of alliance members [10]. The mechanism of learning also guides the development, evolution, and application of dynamic capabilities [11].

Knowledge acquisition capability. No alliance member can solve all the problems that arise during innovative development by depending on its own knowledge; thus, all members should acquire new knowledge from external cooperative partners and incorporate it into their own knowledge stocks, as this is necessary for the maintenance of competitiveness.

Knowledge sharing capability. In the context of knowledge sharing, the knowledge generated during knowledge creation activities is directly integrated; thus, this knowledge is transferred from knowledge stocks to knowledge integration.

Knowledge absorption ability. Absorption capacity is the ability to recognize the value of external information and absorb it. Alliance members with greater absorption capacity exhibit stronger learning and dynamic capabilities and are better able to convert external knowledge into internal knowledge, thereby improving performance; however, firms with weaker absorption ability face severe challenges [12].

The ability to explain knowledge. In the internal environment of an IURCIA, the ability to explain knowledge enables alliance members to comprehend new knowledge, which helps drive the innovative use of existing knowledge and directly improves performance in new product development.

Efficient decision-making ability. In the context of decision-making, alliance members evaluate the risks and performance associated with alliance admission and the effects of the external environment [9], formulate action plans and adjust their alliance mode, aiming to fully exploit the opportunity for knowledge sharing and alleviate the effects of negative factors.

The ability to revolutionize and integrate knowledge. The ability to revolutionize is the third key element of dynamic ability, and it consists of knowledge integration, knowledge exploration, and knowledge innovation. Members with revolutionary capacity can effectively and promptly change their form of cooperation, create, update and reallocate corporate abilities, and develop coordination technology in response to an alliance's action decisions [9]. Successful revolutionization facilitates the coordinated development of a dynamic environment among the members within an alliance, the full utilization of opportunities and knowledge with other members, and the enhancement of competitive advantage. Moreover, the strength of a member's ability to revolutionize also determines its profit level [9].

Integration capability. Knowledge integration can become a source of new knowledge [13] and serve as a platform that reaches a new field of competition [14]. Moreover, through knowledge integration, alliance members can identify gaps in their knowledge resources and realize the necessity of obtaining innovative knowledge.

Exploration capability. When the internal knowledge resources of alliance members are insufficient to solve problems through knowledge innovation, external knowledge resources play an important role in innovation. Knowledge innovation is also a kind of new knowledge since innovation in a competitive environment leads to new knowledge and experiences.

The ability to apply knowledge. When faced with novel problems during new product development, members should use their existing knowledge to create new applications to solve these problems.

*(3) The Added Value of Knowledge*. A direct embodiment of the knowledge management effect is the knowledge state of an enterprise. Since knowledge sharing is a core element of knowledge management, the direct result of IURA knowledge sharing is an improved knowledge state and the ability to preserve knowledge.

Knowledge allocation breadth. Knowledge allocation breadth reflects the number of skill types and specialties possessed by an enterprise [15]. After joining an IURCIA, an enterprise, through knowledge sharing, enters a new technological field to acquire new knowledge and skills that it lacks and urgently needs to learn. Moreover, universities and institutes study and develop new skills in new fields according to their actual demands. An increment in the knowledge allocation breadth of the enterprises in an IURA suggests that the corresponding amount of knowledge has been grasped by its members.

Knowledge allocation depth. Knowledge allocation depth reflects the degree to which an enterprise grasps a given set of knowledge [15]. Alliance members explain and share self-possessed knowledge and, in this process, further understand and apply their original knowledge. Furthermore, enterprises cooperate with researchers from universities and institutes, intensify their knowledge cognition, and accelerate knowledge conversion.

Knowledge stocks. All the members of an alliance can obtain additional external knowledge resources, collaborate on new knowledge with other members, increase their knowledge stocks, and maintain competitiveness. For enterprises, the relevant economic indices include increased profit and the reduction of product innovation costs. For universities and institutes, the relevant economic indices include increases in transverse research investment, increases in the number of patents, and the promotion of achievement conversion efficiency.

This study was based on dynamic capability theory, the collaborative innovation within IURAs, and the knowledge sharing performance evaluation indices summarized in Table 1. We built an IURA knowledge sharing performance evaluation system involving 4 first-level indices (the ability to identify opportunities, the ability to seize opportunities, the ability to revolutionize and integrate knowledge, and the added value of knowledge) and 24 second-level indices. The index system is shown in Table 2.

### 2.2. Questionnaire Design and Measures

Regarding the IURA knowledge sharing performance evaluation indices, 15 questions were designed, including 14 questions about knowledge sharing performance evaluation and 1 question about knowledge sharing performance scoring. The indices were evaluated using a Likert-type scale that ranged from 1 to 5; the highest and lowest scores were 0.9 and 0.1, respectively. Scores 1–5 corresponded to “totally true,” “true,” “neutral,” “false,” and “totally false,” respectively. To evaluate IURA knowledge sharing performance, we had to acquire quantitative results on the effect of knowledge conversion. The output layer consisted of numerical values from 0 to 100, and a value closer to 100 indicated that the knowledge sharing performance was relatively good while a value closer to 0 meant that the performance was relatively bad.

The size and quality of samples used determine the effectiveness of predictions made using the BPNN. We sought to prevent low modeling accuracy stemming from poor sample quality and small sample size and to improve the predictive power of our model. Therefore, we selected managers from 10 members of 5 IURAs. All the managers involved in the questionnaire had at least 5 years of working experience in their positions and deeply understood the research, production, and profit of their own organizations. We questioned 100 managers by visiting or emailing them and modified our questionnaire according to each alliance's actual situation. Eighty-four questionnaires were obtained.

## 3. PSO-BPNN-Based Performance Evaluation Model of Knowledge Sharing in IURAs

BPNN is a multilayer feedforward NN that allows the error to propagate backward while the signal propagates forward [16], and it can simulate the relationship between any type of nonlinear input and output [17].

Inside a BPNN as shown in Figure 1, there are many neurons that can be trained to map the input to the output [16]. The structure of this NN includes an input layer, a hidden layer (middle layer), and an output layer [18]. The performance (e.g., convergence) of the network is very sensitive to the connection weights and thresholds between neurons in adjacent layers. An improper setting of these parameters can severely affect network performance, and some extreme points may even be generated; this leads to local optimal solutions for the network and thus impacts network prediction accuracy [19]. The training and learning processes of the NN are complex and easily lead to over learning [17].

The PSO algorithm mimics the flight and foraging patterns of birds and performs an adaptive probabilistic optimization search [20]. As a highly efficient optimization algorithm, PSO is simple in principle and mechanism, evolving to a global optimal solution without the need for gradient information. This PSO algorithm has only a few parameters, is easy to implement, and is efficient in operation [21]. In relation to addressing the deficiencies of NNs, the PSO algorithm can be used to optimize the structure, learning rules and weights of NNs to improve their learning accuracy and speed [22]. The PSO algorithm includes many processes, such as fitness calculations, initialization, and fitness updating, designed to identify the particle with the optimal position as the solution to the focal problem [23]. A BPNN optimized based on the PSO algorithm has better network approximation properties [24].

(1) The original data are preprocessed, and the resulting data are used as the input values of the NN.
(2) The values of the parameters, such as the population size, variable range, inertia weight, and learning factor, are set, and a group of particles uniformly distributed in the given optimization space (given the particle positions and velocity information) is randomly initialized [25].
(3) The fitness function is determined.
The training error precision *E* is used as an evaluation index of the particle search performance to guide the population search.
  (1) $$\begin{array}{c} \text{fitness}=\frac{1}{1+E}. \end{array}$$
(4) The current fitness of each individual particle in the swarm is compared with its extremum before the iteration, and if the former is better than the latter, the individual extremum is updated. The global extremum is the individual extremum with the best fitness among all the individual extrema. The weight and connection structure of the NN corresponding to the global extremum are the current optimal solutions of the particle swarm [26].
  (2) $$\begin{array}{c} v_{i+1}\left(t+1\right)=\omega v_{i}\left(t\right)+c_{1}r_{1}\left({\text{pbest}}_{i}\left(t\right)-x_{i}\left(t\right)\right)+c_{2}r_{2}\left(\text{gbest}-x_{i}\left(t\right)\right),\\ x_{i+1}\left(t+1\right)=x_{i}\left(t\right)+v_{i+1}\left(t+1\right), \end{array}$$
where: pbest is the particle best position; gbest is the swarm best position; *v*_*i*_ is the velocity vector; *x*_*i*_ is the position vector; *c*_*1*_ and *c*_*2*_ are learning factors; *r*_*1*_ and *r*_*2*_ are two random values between 0 and 1.
(5) The PSO-optimized weights and thresholds are substituted into the BPNN. After a risk test, the PSO-optimized NN is trained with the training samples until the error requirement is satisfied, and the construction of the performance sharing evaluation model for IURAs is thus completed.
(6) The processed data are fed into the trained PSO-BPNN, and reverse normalization is applied to the network output results to obtain the predicted value of the knowledge sharing performance of the IURA.

## 4. Results and Discussion

### 4.1. Data Collection

The performance evaluation index system of knowledge sharing in IURAs consisted of 18 items, including 17 input indices and 1 output index. A five-point Likert scale (completely disagree, disagree, barely agree, agree, and completely agree) that ranged from a low score of 0.1 to a high score of 0.9 was used. The knowledge sharing performance of the IURAs needed to be quantified prior to the evaluation. The output value ranged from 0 to 100. The closer the value was to 100, the better the knowledge sharing performance was; moreover, the closer the value was to 0, the worse the knowledge sharing performance was.

The quantity and quality of samples determines the reliability and effectiveness of network predictions. To prevent poor sample quality and low model prediction accuracy and improve model prediction performance, we selected the personnel of IURAs as survey subjects. The respondents of the questionnaire survey all had in-depth knowledge of the production, learning, and R&D of their respective working units. The data were collected from 100 people using a WeChat questionnaire, and the content was scored according to the actual situation of the alliance. In total, 54 valid questionnaires were ultimately obtained after excluding invalid questionnaires.

### 4.2. Performance Evaluation Results of Knowledge Sharing in an IURA

In this study, a PSO-BPNN prediction model of knowledge sharing performance was constructed with 17 performance evaluation indices of knowledge sharing in an IURA as input items and knowledge sharing performance evaluation results as the output item.

First, the PSO-improved NN was implemented using MATLAB (R2018b), and 40 sets of test samples were used to evaluate the knowledge sharing performance of the examined IURAs. Then, the results were compared with those obtained with the traditional BPNN [27]. In this study, the PSO-BPNN prediction model had a training error of 0.0001, a maximum of 950 training steps, a learning rate of 0.1, 10 hidden layer neurons, and a network structure of 17-17-17-1. To ensure that the network converged rapidly and obtained the global optimal solution [28], the parameters of the PSO algorithm shown in Table 3 were used in this study. There were 17, 17, and 1 nodes in the input layer, hidden layer, and output layer of the BPNN, respectively.

The effects of PSO parameter selection on the predicted values of the PSO-BPNN are summarized as follows:

- Population size *N*: This parameter is related to the size of the problem, which will not converge with either a too large or a too small *N.*
- Inertia weight *ω:* This parameter maintains the motion inertia of the particles, which tends to expand the search space to obtain a better solution. A larger *ω* enables a population to search within a larger range, while a smaller *ω* ensures that the population eventually converges to the optimal position.
- learning factors *c*_*1*_ and *c*_*2*_: These two parameters represent the weights of random acceleration directions that pull each particle toward the pBest and gBest positions, respectively, indicating the “self-learning ability” of the individual and the “social learning ability” of the population. A larger *c*_*1*_ causes all particles to hover too much in the local range, which is not conducive to the global search of the algorithm, while a larger *c*_*2*_ prematurely traps the particles in the local extrema, reducing the accuracy of the solution.

To determine the effectiveness of the PSO-BPNN, we compared the predicted values of the PSO-BPNN with those of the unmodified BPNN. Two indices, i.e., the average relative error (*E*_*MR*_) and the relative error variance (RMSE), were used to evaluate the performance of the prediction model. The robustness of the NN model was measured with the correlation coefficient *R*^*2*^. The smaller the relative error value in equation (3) was, the more accurate the predicted value. The closer the *R*^*2*^ in equation (5) was to 1, the higher the correlation, and the closer the predicted value was to the target value.

(3) $$\begin{array}{c} E_{MR}=\left[\sum_{i=1}^{m}\frac{\left|y_{i}-f\left(x_{i}\right)\right|/y_{i}}{m}\right]\times 100\%, \end{array}$$

(4) $$\begin{array}{c} \text{RMSE}=\sqrt{\frac{1}{N}\sum_{i=1}^{N}{\left(y_{i}-f\left(x_{i}\right)\right)}^{2}}, \end{array}$$

(5) $$\begin{array}{c} R^{2}=1-\left(\frac{\sum_{i=1}^{N}{\left(f\left(x_{i}\right)-y_{i}\right)}^{2}}{\sum_{i=1}^{N}{\left(f\left(x_{i}\right)\right)}^{2}}\right), \end{array}$$

where *y*_*i*_ is the measured value of the test sample and *f*(*x*_*i*_) is the predicted value of the PSO-BPNN.

Figures 2to 6 show the predicted values of the BPNN and PSO-BPNN. As shown in Figure 2, the average fitness after 60 generations of evolution is optimal.  Figure 3 shows that the predicted value of the PSO-BPNN is closer to the experimentally measured value than the predicted value of the BPNN. As shown in Figure 4, the relative error of the PSO-BPNN is lower than that of the BPNN. The performance of the PSO-BPNN and BPNN is presented in Figures 5 and 6. To comprehensively compare the performance of the PSO-BPNN and BPNN, we compared the two models in terms of the number of iterations, error, and NN robustness, and the results are listed in Table 4. Both the *E*_*MR*_ and RMSE of the PSO-BPNN test model are smaller than those of the BPNN. The structure, learning rule, weights, and thresholds of the BPNN optimized by the PSO algorithm are reasonable, and the corresponding predicted results are better than those of the BPNN.

## Figures and Tables

**Figure 1:** Structural system of the BP neural network.

**Figure 2:** Average fitness variation curve with the number of evolutionary generations.

**Figure 3:** Comparison of the predicted values of the BP neural network and the PSO-BP neural network.

**Figure 4:** Comparison of the relative errors of the predicted values of the BP neural network and the PSO-BP neural network.

**Figure 5:** BP neural network performance.

**Figure 6:** PSO-BP neural network performance.

**Table 1:** Knowledge sharing performance evaluation indices and appearance frequency.

Evaluation index	Appearance frequency
Knowledge acquisition capability	14
Communication capability	13
Incentive system	9
Cultural compatibility	9
Knowledge absorption capability	8
Knowledge sharing capability	8
Knowledge stock level	7
Knowledge innovation capability	4
Knowledge application capability	4
New product sales	4
Knowledge discovery capability	2
Knowledge modification capability	2

**Table 2:** The IURA knowledge sharing performance evaluation indices.

Total index	1st-level index	2nd-level index
Knowledge sharing performance evaluation index	Ability to identify opportunities a1	Knowledge lever b1
		Ability to perceive opportunities b2
		Ability to create opportunities b3
		Ability to adapt b4
	Ability to seize opportunities a2	Reaching a consensus b5
		Learning ability b6
		Knowledge acquisition ability b7
		Knowledge sharing ability b8
		Efficient decision-making ability b9
		Knowledge absorption ability b10
		The ability to explain knowledge b11
	Ability to revolutionize and integrate knowledge a3	Integration capacity b12
		Exploration capacity b13
		Innovation capacity b14
		Knowledge application capacity b15
	Added value of knowledge a4	Knowledge allocation breadth b16
		Knowledge allocation depth b17
		Knowledge stock b18
		Knowledge preservation capacity b19
		Achievement conversion improvement b20
		Increase in transverse research expenses b21
		Increase in number of patents b22.
		Profit from innovative products b23
		Cost reduction b24

**Table 3:** PSO parameters.

Population size	Maximum inertia weight	Minimum inertia weight	Learning factor 1	Learning factor 2
20	0.9	0.3	2	2

**Table 4:** Predictive performance comparison of the BP neural network and the PSO-BP neural network.

Neural network	Number of iterations	Maximum relative error (%)	Minimum relative error (%)	Average relative error (%)	Average relative error variance	*R* ^*2*^
BP	2000	13.41	0.13	5.04	5.38	0.998223
PSO-BP	150	1.03	0.0198	0.38	0.46	0.999987

## Data Availability

No data were used to support this study.
